RETRACTED

# Epiploic Appendagitis Clinically Masquerading as an Acute Diverticulitis

**DOI:** 10.7759/cureus.20188

**Published:** 2021-12-05

**Authors:** Razan A Khafaji, Hussain S Ghandourah, Sarah K Altamimi, Afnan A Alwarthan, Renda A Alhabib, Mazen N Alaiyar, Ibrahim A Alomar, Meshari I Alayshan, Mohammed S Almasoudi, Hashem A Jaml Allil, Shahad Z Munshi, Sarah K Aljamri, Basil S Bagadeem, Motaz S Attar, Faisal Al-Hawaj

**Affiliations:** 1 College of Medicine, King Abdulaziz University, Jeddah, SAU; 2 College of Medicine, Maastricht University, Maastricht, NLD; 3 College of Medicine, Arabian Gulf University, Manama, BHR; 4 College of Medicine, King Saud bin Abdulaziz University for Health Sciences, Riyadh, SAU; 5 College of Medicine, Qassim University, Qassim, SAU; 6 College of Medicine, AlMaarefa University, Riyadh, SAU; 7 College of Medicine, Jouf University, Al-Jawf, SAU; 8 College of Medicine, Umm Al-Qura University, Mecca, SAU; 9 College of Medicine, Ibn Sina National College for Medical Studies, Jeddah, SAU; 10 College of Medicine, Imam Abdulrahman Bin Faisal University, Dammam, SAU; 11 College of Medicine, King Saud Bin Abdulaziz University for Health Sciences, Jeddah, SAU

**Keywords:** case report, computed tomography, epiploic appendagitis, acute diverticulitis, abdominal pain

## Abstract

Acute diverticulitis is a prevalent surgical condition that typically presents with lower abdominal pain and tenderness. However, the clinical and laboratory findings of diverticulitis are non-specific and other conditions may give similar manifestations. We present the case of a middle-aged woman with a left lower quadrant abdominal pain and fever of three days duration. On examination, she had tachycardia and localized tenderness in the left iliac fossa with rebound tenderness. There were no signs of peritonitis, including the rigid abdomen and decreased bowel sounds. The laboratory findings were suggestive of an inflammatory or infectious process. A computed tomography scan of the abdomen demonstrated a fat-density lesion anterior to the descending colon representing epiploic appendagitis. The patient was managed conservatively with non-steroidal anti-inflammatory drugs (lornoxicam 8 mg). The patient experienced gradual improvement and was discharged after four days of hospitalization. No surgical intervention was needed. The case highlighted the importance of considering epiploic appendagitis in the differential diagnosis of acute diverticulitis. An accurate diagnosis will prevent the patient from having unnecessary surgeries as conservative management is often sufficient in patients with epiploic appendagitis.

## Introduction

Colonic diverticular disease is a significant cause of hospitalization and a major contributor to healthcare costs. However, more than 95% of patients with diverticular disease do not develop acute diverticulitis [1]. The clinical manifestation of diverticulitis includes left-sided abdominal pain with nausea and vomiting. However, the clinical diagnosis of acute diverticulitis often lacks accuracy. The incorrect diagnosis of acute diverticulitis reaches up to 65% [2]. A computed tomography scan of the abdomen provides an accurate diagnosis of acute diverticulitis promptly. The differential diagnoses of acute diverticulitis include a wide range of conditions, including urinary stone disease, small intestinal obstruction, acute cholecystitis, acute appendicitis, and ovarian pathologies [3]. It is crucial to make the correct diagnosis of the acute diverticular disease since some benign conditions may have a similar clinical manifestation and do not require any surgical intervention. Here, we present the case of a middle-aged woman with acute appendagitis clinically masquerading as acute diverticulitis.

RETRACTED

## Case presentation

We present the case of a 51-year-old woman who presented to the emergency department complaining of abdominal pain for three days. The pain was localized in the left lower quadrant and was non-radiating. She reported that the pain was constant and was stabbing in nature. She scored the pain as 7 out of 10 on the severity scale. The pain was exacerbated by food intake and was not related to posture or movement. She attempted over-the-counter analgesics that resulted in mild improvement in her pain. The pain was associated with a low-grade fever that measured 37.9℃. The patient reported that she had decreased bowel motion for the last one week. She reported no history of vomiting or abdominal distension. No history of previous similar pain episodes.

The past medical history for the patient was remarkable for diabetes mellitus and gastroesophageal reflux disease. The patient had obesity with a body mass index of 32 kg/m2. She underwent mastectomy for invasive ductal carcinoma. Her medications included metformin 1000 mg and omeprazole 40 mg daily. No history of allergies. She was a heavy smoker with 30 pack-years of smoking. No history of alcohol intake. The family history was remarkable for inflammatory bowel disease.

Upon examination, the patient appeared in distress due to the pain. The vital signs showed tachycardia (122 bpm), normal temperature (37.8℃), normal respiratory rate (15 bpm), and maintained blood pressure (110/70 mmHg). Abdominal examination revealed a localized tenderness and guarding in the left iliac fossa with rebound tenderness. No palpable masses were noted. Auscultation of the abdomen revealed bowel sounds of normal intensity and frequency. Examination of other systems was non-contributory.

RETRACTED

Initial laboratory investigations were suggestive of the inflammatory process. They revealed leukocytosis (13,000/μL) and elevated C-reactive protein (15 mg/dL), and erythrocyte sedimentation rate (25 mm/hr). The renal and hepatic profiles were within the normal ranges (Table 1). The urinalysis findings were normal.

**Table 1:** Summary of the results of laboratory findings

Laboratory Investigation	Unit	Result	Reference Range
Hemoglobin	g/dL	14.1	13.0–18.0
Leukocytes	1000/mL	13.0	4.0–11.0
Platelet	1000/mL	440	140–450
Erythrocyte Sedimentation Rate	mm/hr.	25	0–20
C-Reactive Protein	mg/dL	15.0	0.3–10.0
Total Bilirubin	mg/dL	0.8	0.2–1.2
Albumin	g/dL	4.5	3.4–5.0
Alkaline Phosphatase	U/L	49	46–116
Gamma-glutamyltransferase	U/L	17	15–85
Alanine Transferase	U/L	18	14–63
Aspartate Transferase	U/L	15	15–37
Blood Urea Nitrogen	mg/dL	10	7–18
Creatinine	mg/dL	0.7	0.7–1.3
Sodium	mEq/L	138	136–145
Potassium	mEq/L	3.9	3.5–5.1
Chloride	mEq/L	104	98–107

The clinical findings conferred the diagnosis of acute diverticulitis. The patient was kept nil per mouth for bowel rest. Intravenous hydration, analgesics, and broad-spectrum antibiotic (ceftriaxone) were administered. The patient was planned for laparoscopic surgery. However, an abdominal computed tomography scan with intravenous contrast was performed in order to identify the presence of any intra-abdominal collection. The scan demonstrated the presence of a fusiform lesion of hypoattenuation located anterior to the descending colon with a prominent rim of hyperdense halo. Minimal stranding of the surrounding fat planes was observed. There was no evidence of colonic diverticular disease. No pneumoperitoneum of free fluid was noted. Such findings conferred the diagnosis of epiploic appendagitis (Figure 1-2).

**Figure 1:** Axial CT image of the abdomen demonstrates an oval-shaped fat-density structure with hyperdense rim (arrow) representing epiploic appendagitis. CT: computed tomography

**Figure 2:** Coronal CT image demonstrates a fusiform fat-density lesion (arrow) adjacent to the descending colon representing epiploic appendagitis. CT: computed tomography

Since epiploic appendagitis is a self-limiting condition, the patient was kept on intravenous lornoxicam 8 mg. The patient responded well to this non-steroidal inflammatory drug and she reported gradual resolution of her pain over three days. The patient was discharged after four days of hospitalization. After three months of follow-up, the patient remained asymptomatic.

## Discussion

We present the case of a rare case of epiploic appendagitis clinically masquerading as acute diverticulitis. Epiploic appendagitis is a rare inflammatory condition caused by ischemic infarction of fat-filled serosa-covered structures of the colon. Epiploic appendagitis is a relatively rare condition and might be a great mimicker of acute appendicitis or diverticulitis, as in the present case. The annual incidence of epiploic appendagitis is less than 10 cases per million [4]. Further, a prior study revealed that 1% of suspected acute appendicitis is diagnosed as epiploic appendagitis [5].

RETRACTED

In contrast to our case, epiploic appendagitis tends to develop in men. The mean age of diagnosis is 40 years and it frequently occurs in the second to fifth decades of life. The pathogenesis of epiploic appendagitis involves an acute torsion or spontaneous thrombosis of its draining vein [6].

Regarding the clinical manifestation of epiploic appendagitis, it classically presents with acute onset of lower abdominal pain. The site of the pain corresponds to the location of the epiploic appendage which may occur in any segment of the colon. On physical examination, a localized tenderness may be appreciated [7]. The laboratory findings are non-specific and may suggest an inflammatory response. In the present case, the patient had localized left iliac fossa tenderness with elevated white cell counts, C-reactive protein, and erythrocyte sedimentation rate mimicking the classic presentation of acute diverticulitis.

The accurate diagnosis of epiploic appendagitis can be reached using cross-sectional imaging studies. The computed tomography scan can make the diagnosis readily. It demonstrates a small, oval-shaped, fat-attenuation lesion adjacent to the colon with stranding of the surrounding fat. The lesion may have a central dot within the appendage that corresponds to the thrombosed central draining vein, which is known as the dot sign [8]. In the present case, there was no evidence of colonic outpouching with colonic wall thickening and enhancement to suggest acute diverticulitis.

Considering the rarity of the condition, there are no established guidelines about the optimal management approach for patients with epiploic appendagitis. However, the limited data from case reports suggest that patients can be managed conservatively with anti-inflammatory medications and if needed a short course of opioids [6,8]. The medical treatment does not alter the course of the disease, but it results in symptomatic improvement. If the conservative treatment failed to result in improvement, surgical ligation of the appendages can be performed. In the present case, the use of a non-steroidal inflammatory drug was sufficient to relieve the symptoms [7].

RETRACTED

## Conclusions

Epiploic appendagitis is a self-limited condition that can be a great mimicker of acute diverticulitis. Clinicians should keep this diagnosis in mind when they encounter a patient with acute lower abdominal pain. Accurate diagnosis of epiploic appendagitis allows the patient to avoid unnecessary abdominal surgeries. Conservative management with anti-inflammatory medications is usually sufficient.
